The article "Epitopes screening and vaccine molecular design of SADS-CoV based on immunoinformatics" was retracted in 2023. Reason: concerns about the authorship.

# Epitopes screening and vaccine molecular design of SADS-CoV based on immunoinformatics

**DOI:** 10.3389/fvets.2022.1080927

**Published:** 2023-03-02

**Authors:** Shinian Li, Yaping Chen

**Affiliations:** College of Animal Science and Veterinary Medicine, Heilongjiang Bayi Agricultural University, Daqing, Heilongjiang, China

**Keywords:** Swine acute diarrhea syndrome coronavirus (SADS CoV), spike protein, immunoinformatics, epitope vaccines, antigen epitope

## Abstract

The regional outbreak of the Swine acute diarrhea syndrome coronavirus (SADS-CoV) has seriously threatened the swine industry. There is an urgent need to discover safe and effective vaccines to contain them quickly. The coronavirus spike protein mediates virus entry into host cells, one of the most important antigenic determinants and a potential vaccine target. Therefore, this study aims to conduct a predictive analysis of the epitope of S protein B cells and T cells (MHC class I and class II) by immunoinformatics methods by screening and identifying protective antigenic epitopes that induce major neutralized antibodies and activate immune responses to construct epitope vaccines. The study explored primary, secondary, and tertiary structures, disulfide bonds, protein docking, immune response simulation, and seamless cloning of epitope vaccines. The results show that the spike protein dominant epitope of the screening has a high conservativeness and coverage of IFN-γ, IL-4-positive Th epitope, and CTL epitope. The constructed epitope vaccine interacts stably with TLR-3 receptors, and the immune response simulation shows good immunogenicity, which could effectively activate humoral and cellular immunity. After codon optimization, it was highly likely to be efficiently and stably expressed in the *Escherichia coli* K12 expression system. Therefore, the constructed epitope vaccine will provide a new theoretical basis for the design of SADS-CoV antiviral drugs and related research on coronaviruses such as SARS-CoV-2.

## 1. Introduction

Swine acute diarrhea syndrome (SADS) is a highly contagious, acute, and fatal respiratory and gastrointestinal infectious disease of pigs caused by Swine acute diarrhea syndrome coronavirus (SADS-CoV) (1). The first outbreak occurred in Qingyuan district, Guangdong Province, China, in 2017, causing severe economic losses to the pig industry in the region (2). The clinical symptoms of diseased pigs were similar to those of other porcine intestinal coronaviruses, and the clinical manifestations were mild diarrhea in infected sows (3). Infected newborn piglets within 5 days of age suffer from acute diarrhea and vomiting, resulting in acute death, and the mortality rate can be as high as 90% (4). Given is that SADS-CoV was a newly emerged coronavirus in pigs in China, the current understanding and research on SADS-CoV were still shallow. No commercial vaccine was available, bringing challenges to its prevention and control. Therefore, the effect of its antigen characteristics and antigen variation on the host protective immune response needs further clarification.

The article "Epitopes screening and vaccine molecular design of SADS-CoV based on immunoinformatics" was retracted in 2023. Reason: concerns about the authorship.

Viral antigens, including S protein, have multiple epitopes that have immunoprotective effects and induce the neutralization of antibodies (such as antibodies that inhibit virus replication), effector T cells that inhibit or kill infected cells and assist immune balance response (5). However, the immune response induced by most epitopes does not have the function of neutralizing or inhibiting virus replication (6). On the contrary, it might induce an imbalance of cellular immune response and aggravate inflammatory response, with negative risks such as immunopathological damage and antibody-dependent enhancement (ADE), It might even attenuate the immune protective effect of immunoprotective epitopes (7). Immunoinformatics is used to predict antigenic epitopes' characteristics from the gene sequence source, screen the results, and analyze and identify the dominant epitopes with immune protection (8). It could effectively improve protective antibody affinity and cellular immune balance, triggering the immune system to develop immunity to viruses. Therefore, dominant viral epitopes are ideal candidates for vaccine construction (9).

The total length of the SADS-CoV genome is about 27.17 kb, encoding four major structural proteins, including spike protein (S), nucleocapsid protein (N), membrane protein (M), and small membrane protein (E) (10). Among them, the S protein of SADS-CoV and other coronavirus is a key target for vaccine and antiviral drug development (11). Vaccines of S protein could induce the body to produce neutralizing antibodies among all structural proteins located on the surface of virions, cell attachment, receptor-bound, interspecies transmission, mediated viral invasion, and infection. It was the main antigen component responsible for induced host immune response and protected immunity against viral infection (12). Therefore, the full-length trimeric S protein usually has high immunogenicity; however, vaccines with full-length S proteins could also induce harmful immune responses that lead to liver damage in vaccinated animals or aggravated infection after homologous virus infection (13). To avoid toxic side effects and enhance the immune effect of the vaccine, in this study, based on immunoinformatics, we screened, identified, and constructed epitope vaccines for the dominant protective epitopes of SADS-CoV S protein and used molecular docking analysis, immune simulation prediction and *silico* clone of epitope vaccine. The purpose was to provide a new method for the design of the SADS-CoV epitope vaccine and a theoretical basis and data support for developing the SADS-CoV epitope vaccine.

The article "Epitopes screening and vaccine molecular design of SADS-CoV based on immunoinformatics" was retracted in 2023. Reason: concerns about the authorship.

## 2. Materials and methods

The workflow summarizing the procedures for the epitope-based candidate vaccine prediction is shown in Figure 1.

**Figure 1:** Descriptive workflow for the epitope-based candidate vaccine prediction.

### 2.1. Determination of candidate vaccine strains of SADS-CoV

From the NCBI (https://www.ncbi.nlm.nih.gov/protein) database, we collected 31 amino acid sequences of SADS-CoV S protein in fasta file format and used this as a template. The MEGA 7.0 software was used to analyze the sequence conservation, and then the WebLogo server (http://weblogo.berkeley.edu/logo.cgi) was used to visualize the obtained comparative data set.

### 2.2. Prediction and screening of epitopes

The PEPTIDES (http://imed.med.ucm.es/Tools/antigenic.pl) and ABCpred server (https://webs.iiitd.edu.in/raghava/abcpred/index.html) were used to predict candidate linear B lymphocyte epitopes of the SDS-CoV S protein. The former antigenic peptides are determined used the method of Kolaskar and Tongaonkar. Predictions are based on a table that reflects the occurrence of amino acid residues in experimentally known segmental epitopes. Segments are only reported if the have a minimum size of 8 residues. The reported accuracy of method is about 75%, the latter ABCpred is a recursive neural network based learned algorithm with a default threshold of 0.51 and a tableau length of 16, and its accuracy is 65.93% (14, 15). The NetMHCIIpan-4.0 server (https://services.healthtech.dtu.dk/service.php?NetMHCIIpan-4.0) was used to predict MHC-II epitopes to select different alleles. The NetMHCIIpan-4.0 server uses the artificial neural network (ANN) to predict the binding of peptides to any MHC II molecule of known sequence. Under the default threshold, different alleles are used to screen, and finally the strong binding sequence with a percentage greater than 10% is selected (16). Helper T cell Th1 activates macrophages by releasing (interferon γ, IFN-γ), recognizes and clears intracellular pathogens; helper T cell Th2 mainly secretes cytokines (interleukin 4, IL-4), which can promote antigen presentation Cell proliferation and differentiation play a key role in various biological activities. Therefore, The combination potential of epitope and MHC-II was realized through the EpiTOP server (http://www.ddg-pharmfac.net/epitop/) evaluation. IFN-γ inducible antigen and non-IL-4 inducible antigen epitopes pass through the IFNepitope server (http://crdd.osdd.net/raghava/ifnepitope/) and IL4pred server (http://crdd.osdd.net/raghava/il4pred/) forecast (17–19). MHC-I combined CTL epitope prediction by NetMHCpan4.1 server (https://services.healthtech.dtu.dk/service.php?NetMHCpan-4.1) and IEDB server (http://tools.iedb.org/mhci/). The screened method of NetMHCpan4.1 server was the same as that of NetMHCIIpan-4.0 server. The IEDB server uses a consensus recommendation method consisted of ANN, SMM and CombLib, Select different alleles at other default thresholds with lengths of 15 (16, 20). All predicted epitopes were determined by the IEDB server (http://tools.iedb.org/immunogenicity/). An immunogenicity test was carried out, which is non-toxic, through the ToxinPred server (https://webs.iiitd.edu.in/raghava/toxinpred/design.php). Epitopes with immunogenicity score >0.1 and non-toxic were selected as the final prediction (21). At the same time, Pymol software was used to mark the spatial position of each dominant epitope in the tertiary structure of S the (PDB ID:6M39) protein.

The article "Epitopes screening and vaccine molecular design of SADS-CoV based on immunoinformatics" was retracted in 2023. Reason: concerns about the authorship.

### 2.3. Identification of protective epitopes and evaluation of antigenic epitope conservation

To further select the dominant epitope regions for analysis by compared B cell epitopes, Th epitopes and CTL epitopes generated by the server, and the best fragment with high overlap was found. Dominant epitopes were then assessed by the conservation analysis tool on the IEDB server (http://tools.iedb.org/conservancy/), According to the determined candidate epitopes and 31 different SADS-CoV S protein sequences, the conservation of antigen epitopes was analyzed (22).

### 2.4. Construction of candidate vaccines and prediction of antigenicity, sensitization, solubility, and physicochemical properties

Vaccine amino acid sequences were constructed used the above selected CTL, HTL and B lymphocyte dominant epitopes, with the different dominant epitopes linked in tandem using flexible linkers. CTL epitope used GGPPG, HTL epitope used AAY, and B lymphocyte epitope used KK. In order to improve the immunogenicity of candidate vaccines, β- Defensin I, as an immune enhancer, is connected to the N-terminal of the construct through EAAAK linkers (23). Through the ANTIGENpro server (http://scratch.proteomics.ics.uci.edu/) and VaxiJen v2.0 server (http://www.ddg-pharmfac.net/vaxijen/VaxiJen/VaxiJen.html) for the final built antigenicity analysis of candidate vaccines (24, 25); AllerTOPv2.0 server (http://www.ddg-pharmfac.net/AllerTOP), for the final built allergenicity analysis of candidate vaccines (26); SOLpro server (http://scratch.proteomics.ics.uci.edu/explanation.html#SOLpro) for the final built solubility analysis of candidate vaccines (27). In addition, the final candidate vaccine should also pay attention to its physical and chemical properties. Therefore, used the ExPASy Server (https://web.expasy.org/protparam/) for the physicochemical properties of the candidate vaccine were analyzed (28).

The article "Epitopes screening and vaccine molecular design of SADS-CoV based on immunoinformatics" was retracted in 2023. Reason: concerns about the authorship.

### 2.5. Candidate vaccine secondary and tertiary structure modeling, refining, and disulfide engineering

Candidate vaccine used the PSIPRED4.0 server (http://bioinf.cs.ucl.ac.uk/psipred) and SOPMA server (http://npsa-prabi.ibcp.fr/cgi-bin/npsa_automat.pl?page=npsa_sopma.html) completes the prediction of the secondary structure of the final candidate vaccine (14, 29). The trRosetta server (https://yanglab.nankai.edu.cn/trRosetta/) completes the prediction of the tertiary structure of the final candidate vaccine (30). At the same time, used the Galaxy-WEB server (https://galaxy.seoklab.org/cgi-bin/submit.cgi?type=REFINE) the quality of the model was improved, and the coarse structure in the model was optimized in this process (31). For this purpose the EBI-PDBSum server (http://www.ebi.ac.uk/thornton-srv/databases/pdbsum/Generate.html) a Ramachandran diagram was generated to evaluate the quality of the model before and after optimization (32). Before proceeding to the next step, it was necessary to improve the stability of the candidate vaccine model. Therefore, used the DisulfidebyDesign2.0 server (http://cptweb.cpt.wayne.edu/DbD2/index.php) performs disulfide engineered on candidate vaccines (33). After that used the ProSA-web server (https://prosa.services.came.sbg.ac.at/prosa.php) was used to perform global detection on the model (34).

### 2.6. Tertiary epitope prediction and protein docking analysis

ElliPro server (http://tools.iedb.org/ellipro/) conformational B-cell epitopes for prediction of vaccine protein tertiary structure (35). Meanwhile, protein interactions are important for understanding cell function and tissue structure. Molecular docking was a method to predict the interaction between a receptor and a ligand in a stable conformation. Therefore, used the PyDockWEB server (https://life.bsc.es/pid/pydockweb) for the interaction between TLR3 (PDB ID: 2A0Z) as receptor and protein vaccine as ligand is predicted (36). LigPLot+ was used to determine the amino acid residues with hydrogen bonds and hydrophobic interactions after docking.

### 2.7. Immune simulation, codon optimization, and silico cloning

Immunoresponse analysis of the final constructed candidate vaccine by the C-ImmSim server (https://150.146.2.1/C-IMMSIM/index.php) was performed to evaluate the immunogenicity characteristics of the candidate vaccine (37). The immunization process was conducted every 7 days, 3 times in total, and the time steps were set as 1, 20, and 40 (each time step was 8 h), where default remained simulation parameters. Back translation of the candidate vaccine's amino acid sequence was conducted on the Gene infinity server (http://www.geneinfinity.org/sms/sms_backtranslation.html) (38). The Codon Adaptation Index (*CAI*) and GC content of optimized DNA were assessed by the GenScript server (https://www.genscript.com/tools/rare-codon-analysis) (Genscript Biotech Corporation, China). Finally, the candidate vaccine sequence was inserted into the pET-30a (+) vector by the SnapGene tool.

The article "Epitopes screening and vaccine molecular design of SADS-CoV based on immunoinformatics" was retracted in 2023. Reason: concerns about the authorship.

## 3. Result

### 3.1. Conservative analysis of SADS-CoV S protein and determination of vaccine strain

The amino acid sequences of 31 SADS-CoV S proteins downloaded from the NCBI database were analyzed by MEGA 7.0 software. Finally, the relatively conserved SDS-COV S protein (ASK51717.1) was selected as the template for cell epitope prediction. WebLogo server visualized proteins' full-length amino acid sequence on the comparative data set obtained by MEGA 7.0 software. Protein conservation is shown (Figure 2), indicating that the C-terminal amino acid mutation of the S protein is obvious. The N-terminal amino acid sequence is relatively conserved.

**Figure 2:** Results of SADS CoV full length S protein conservation analysis.

### 3.2. Screening of S protein dominant epitopes of SADS-CoV

The overlapping epitope regions of B lymphocyte epitopes screened by PEPTIDES server and ABCpred server are shown (Table 1). The epitopes screened by NetMHC II panv4.0 EL server, and then, overlapped epitopes were evaluated by the EpiTOP server for binding potential, further obtaining IFN-γ and non-IL-4 inducible antigen epitopes. The Th epitopes of MHC class II molecules are shown (Table 2). NetMHCpan4.1 server and IEDB server screened overlapping regions of CTL binding epitopes, CTL epitopes are shown (Table 3). In the epitope screening strategy of this study. To make the results reliable and more confident, all predicted dominant epitopes were tested for immunogenicity by IEDB server and its non-toxicity was confirmed by ToxinPred server. The confirmed dominant epitopes are presented in the table by Percent of protein sequence and Minimum identity conservation analysis. The spatial positions of the dominant epitopes are shown (Figure 3).

**Table 1:** Candidate B cell epitopes.

**Name**	**Sequences**	**Length**	**Start position**	**End position**	**Toxin prediction**	**Percent of protein sequence ≦100%/%**	**Minimum identity/%**
B1	NAFECLIN	8	147	154	non-toxin	100.00% (31/31)	100.00%
B2	WYNDLVRIVFPPTV	14	171	184	non-toxin	96.77% (30/31)	92.86%
B3	DFQHLIL	7	316	322	non-toxin	96.77% (30/31)	85.71%
B4	VNRTIVTPYLKPYECF	16	357	372	non-toxin	100.00% (31/31)	100.00%
B5	GDGFCADL	8	531	538	non-toxin	100.00% (31/31)	100.00%
B6	AIEDLLFS	8	675	682	non-toxin	100.00% (31/31)	100.00%
B7	TTPGLCES	8	931	938	non-toxin	100.00% (31/31)	100.00%
B8	TFANVIAVSR	10	975	984	non-toxin	100.00% (31/31)	100.00%

The article "Epitopes screening and vaccine molecular design of SADS-CoV based on immunoinformatics" was retracted in 2023. Reason: concerns about the authorship.

**Table 2:** Candidate Th cell epitopes.

**Name**	**Sequences**	**Allele**	**Start position**	**IFN-γ** **inducer**	**IL-4 inducer**	**Percent of protein sequence ≦100%/%**	**Minimum identity/%**
Th-1	FNTIFSTH RGLSNTT	DRB1_1302; DRB1_0801 DRB1_1301; DRB1_1601	27	Positive	Inducer	100.00% (31/31)	100.00%
Th-2	KLRLFDIP PGVYSNS	HLA-DQA10102-DQB10501 HLA-DPA1*02: 01 DPB1*14: 01 HLA-DPA10401-DPB10901	247	Positive	Inducer	96.77% (30/31)	93.33%
Th-3	VPGFVLRV GRGKAVN	DRB5_0101	347	Positive	Inducer	96.77% (30/31)	93.33%
Th-4	NNTITVK TTPGLCES	DRB1_1501	924	Positive	Inducer	100.00% (31/31)	100.00%
Th-5	NMRVEVE KFQRYVNY	HLA-DPA10202-DPB10402 HLA-DPA10301-DPB10401 HLA-DPA10103-DPB10401 HLA-DPA10201-DPB10101 HLA-DPA10103-DPB10201	1,052	Positive	Inducer	93.55% (29/31)	93.33%

**Table 3:** Candidate CTL cell epitopes.

**Name**	**Sequences**	**Allele**	**Start position**	**Immunogenicity**	**Toxin prediction**	**Percent of protein sequence 100%/%**	**Minimum identity/%**
CTL-1	SVDFNLFNTIFSTH	SLA-1-YDL01	21	0.3763	non-toxin	100.00% (31/31)	100.00%
CTL-2	TNLTWELWIHRKWG	SLA-1-HB02	103	0.7108	non-toxin	100.00% (31/31)	100.00%
CTL-3	PVTNERYTEMPLDH	SLA-6*0104	559	0.1079	non-toxin	100.00% (31/31)	100.00%
CTL-4	IPELNSTFPIEEEF	SLA-1*0201 SLA-1*1301	997	0.3618	non-toxin	93.55% (29/31)	92.86%

**Figure 3:** Epitopes of SADS-CoV Spike protein candidate antigen. Tertiary structure of the spike protein with CTL epitopes marked by red color; HTL epitopes are marked by blue color and IFN-γ epitopes marked by green color; showing their surface positions.

### 3.3. Construction of SADS-CoV S candidate vaccine

Based on the dominant epitopes obtained from the immunoinformatics analysis, a flexible linker tandem candidate vaccine was used to prolong the time of protein action *in vivo*,Effectively avoid the introduction of new bound epitopes. Defensin I plays a role as an immunopotentiator through the N-terminal EAAAK linker, promoting a lasting immune response. AAY and GPGPG linkers enhance the recognition of vaccine subunits and KK connectors to enhance the folding, stability, and expression of proteins. Therefore, the constructed vaccine amino acid sequence was as follows: GIINTLQKYYCRVRGGRCAVLSCLPKEEQIGKCSTRGRKCCRRKKEAAAKFNTIFSTHRGLSNTTAAYKLRLFDIPPGVYSNSAAYVPGFVLRVGRGKAVNAAYNNTITVKTTPGLCESAAYNMRVEVEKFQRYVNYGPGPGSVDFNLFNTIFSTHGPGPGTNLTWELWIHRKWGGPGPGPVTNERYTEMPLDHGPGPGIPELNSTFPIEEEFKKNAFECLINKKWYNDLVRIVFPPTVKKDFQHLILKKVNRTIVTPYLKPYECFKKGDGFCADLKKAIEDLLFSKKTTPGLCESKKTFANVIAVSR. The epitope vaccine kit is shown (Figure 4).

The article "Epitopes screening and vaccine molecular design of SADS-CoV based on immunoinformatics" was retracted in 2023. Reason: concerns about the authorship.

**Figure 4:** SADS-CoV multi-epitope vaccine kit.

### 3.4. Antigenicity, sensitization, solubility, and physicochemical properties analysis of candidate vaccine

ANTIGENpro server and Vaxijenv2.0 server predicted the antigenicity index of candidate vaccine to be 0.892070 and 0.4974, respectively. And the results were far greater than the default threshold of the server, indicating that the constructed vaccine had good antigenicity. In the AllerTOP V2.0 server prediction of vaccine sensitization, the candidate vaccine was found to be non-allergenic. The SOLpro server predicted a solubility probability of 0.924097 at overexpression, much higher than the server's default threshold of 0.5, indicating a high solubility. ExpasyProtparam server forecast results show that: the number of amino acids of candidate vaccine is 308 aa, molecular weight 34.49 ku, theoretical pI 9.61, the estimated half-life was: 30 h (mammalian reticulocytes, *in vitro*), >20 h (yeast, *in vivo*) and > 10 hours (*Escherichia coli, in vivo*). The instability index (II) is computed as 26.43, The instability index (II) was computed to be 72.79, with a grand average of hydropathicity (GRAVY)−0.390. So the server classifies it as a stable hydrophilic protein. The aliphatic chains in the globular protein structure represent the protein's thermal stability. The elevated aliphatic index indicates that the protein is heat-stable.

### 3.5. Candidate vaccine secondary structure prediction

The prediction results of the PSIPRED and SOPMA servers on the secondary structure show that: In the secondary structure of candidate vaccine, the alpha helix is 29.87%, the Extended strand is 22.40%, the Beta turn is 8.12%, and the random coil is 39.61%. The Secondary structure prediction is shown (Figure 5).

**Figure 5:** Secondary structure prediction of SADS-CoV epitopes-based vaccine. Different colors indicate the corresponding information of the secondary structure of the protein.

### 3.6. Modeling, elaboration, and evaluation of candidate vaccine tertiary structure

The results of the best model for the tertiary structure of candidate vaccines predicted by the 3Dpro server are shown (Figure 6F). The results are shown in Figures 6A–E, that is section visualizes predicted 2D information including: Contact map, which displays the predicted probability of residue pairs being in contact, i.e., the distance between their C-beta (C-alpha for Glycine) atoms is less than 8Å. Distance map displays the predicted real distance (4–20 Å) between residue pairs. Orientation maps contains maps of omega (−180°, 180°), theta (−180°, 180°) and phi (0°, 180°). The PROCHECK server generates a Ramachandran diagram (Figure 7A). In the rough model, residues in the most favored regions are 90.3%, 8.5% in the additional allowed regions, 0.8% in generously allowed regions, and 0.4% in the disallowed regions. The Galaxy-Refine server was used to refine the crude model structure in the server-generated five refined models. The parameters of the crude model before refining are GDT-HA (1.0000); RMSD (0.000); MolProbity (1.268); Clash score (3.6); Poorrotamers (00.0); and Rama favored (97.4). After refining, it was confirmed that the first model was the best candidate. The parameters of the model were GDT-HA (0.9440), RMSD (0.430), MolProbity (1.233), Clash score (4.6), Poorrotamers (0.8), and Rama favored (98.7). PROCHECK server generates a Ramachandran diagram (Figure 7C). In the refining model, residues in the most favored regions are 94.2%, 5.4% in the additional allowed regions, 0.0% in the generously allowed regions, and 0.4% in the disallowed regions. For this purpose, Pymol software was used to plot the comparison results, as shown in Figure 7B. To stabilize the protein structure, this study further used the disulfide engineered disulfide by Design 2.0 server to generate disulfide-stabilized proteins. The prediction results show that the B-factor was 0. It was considered that the tertiary structure model of the candidate vaccine after refining was stable enough, and it was not necessary to draw further disulfide bond mutants. Finally, the ProSA web server scored and verified the refined model. The structural accuracy analysis showed that the z value is −3.33 (Figure 7D), and the known-based energy is mostly negative (Figure 7E). The results suggested that the refined model accuracy could meet the requirements for further analysis.

The article "Epitopes screening and vaccine molecular design of SADS-CoV based on immunoinformatics" was retracted in 2023. Reason: concerns about the authorship.

**Figure 6:** Modeling of epitope vaccine tertiary structure. **(A–E)** Omega, Phi, Distance, Theta and Contact parameters of 2D structures; **(F)** Tertiary structure of candidate vaccine, Red: β-Defensin I molecular adjuvant; Yellow: CTL epitopes; Purple: Th epitopes; Green: B cell epitopes; TM-score: 0. 376.

**Figure 7:** Validation of tertiary structure of epitope vaccine. **(A)** Ramachandran plots to validate the tertiary structure; **(B)** For comparison of tertiary protein structure, the crude model and refined model are green and red, respectively; **(C)** The Ramachandran mapping validates the optimized tertiary structure; **(D)** The Z fraction of the ProSA SEB diagram of the refined model is −3.34; **(E)** The quality of the local model is shown by plotting the energy as a function of the position of the amino acid sequence.

### 3.7. Tertiary structure epitope prediction and protein docking

The ElliPro server predicted five B-cell linear epitopes based on the refined tertiary structure model of epitope vaccines: 110–152, 225–272, 44–89, 194–208, and 172–180, the corresponding scores are: 0.744, 0.735, 0.714, 0.696, and 0.617. 7 B-cell conception epitopes, started from the following locations: 48–73, 138–149~151–152~155–167, 193–201, 173~175–180~233–272, 74–86~109–137, 202–206, and 226–232, the corresponding scores are: 0.768, 0.762, 0.751, 0.74, 0.718, 0.637, and 0.629. All scores were above the set threshold of 0.5, confirming that the designed candidate vaccine had good immunogenicity. PyDockWEB server performs protein + protein rigid docking of vaccine ligands and TLR3 receptors. According to the docking result, 101 models were produced, with model name 196 ranking first among all the predicted models from PyDockWEB. The docking result is shown in Figure 8A. The prominent hydrogen bond amino acid residue was locally magnified. The results are shown in Figures 8B, C. LigPLot+ was used to determine the two-dimensional interaction diagram, and the results are shown in Figure 8D. Candidate vaccine ligands and TLR3 receptors had amino acid residues with hydrogen bonds, respectively: Ala405, His460, Ser372, and Ser315. The amino acid residues with hydrophobic interactions are respectively: Thr623, Phe314, Trp429, His312, Asp347, Thr376, Asn373, Asp348, His432, Phe349, Gln352, His316, Trp353, His319, Asp292, Trp296, Lys272, Ala295, Glu456, Asn291, and Asn265.

**Figure 8:** Complexes of candidate vaccine protein docking with human TLR3 receptor. **(A)** Epitope vaccine structure is shown in blue and TLR3 in green; **(B)** Residue of interaction between docking TLR3 and epitope vaccine; **(C)** Local magnification highlights amino acid residues; **(D)** LigPLot+ determined two-dimensional interaction diagram.

### 3.8. Computer simulation of immune response stimulation

C-ImmSim server simulates the candidate vaccine immune response, and the simulation generates significantly higher secondary and tertiary responses than the primary response. Secondary and tertiary reactions show decreased antigen concentrations and increased levels of immunoglobulin activity (IgG1+IgG2, IgM, and IgG+IgM antibodies). In addition, various persistent B cell homotypes were found, while the concentration of adjuvant (TH) and cytokines is also increasing. TH (helper cell) and TC (cytotoxic) cell populations showed similarly higher responses to TC preactivation during vaccination, NK (Natural Killing) and dendritic cell activity were found to be consistent with higher macrophage activity, and high levels of IFN-γ and IL-2 were also triggered in the simulation. Overall, the entire simulated immune response stimulation conforms to the law of inducing an immune response, has good immunogenicity, and can effectively activate humoral and cellular immunity, and the result is shown in Figures 9–11.

The article "Epitopes screening and vaccine molecular design of SADS-CoV based on immunoinformatics" was retracted in 2023. Reason: concerns about the authorship.

**Figure 9:** B cell and Th counts shown *in silico* immune simulation. **(A)** B lymphocytes, total count, memory cells, and sub-divided in isotypes IgM, IgG1 and IgG2; **(B)** Plasma B lymphocytes count sub-divided per isotype (IgM, IgG1 and IgG2); **(C)** B lymphocytes population per entity-state (i.e, showing counts for active, presenting on class-II, internalized the Ag, duplicating and anergic; **(D)** CD4 T-helper lymphocytes count. The plot shows total and memory counts; **(E)** CD4 T-helper lymphocytes count sub-divided per entity-state (i.e., acctive, resting, anergic and duplicating); **(F)** CD4 T-regulatory lymphocytes count. Both total, memory and per entity-state counts are plotted here. Act, active; Intern, internalized the Ag; Pres II, presenting on MHC II; Dup, in the mitotic cycle; Anergic, anergic; Resting, not active.

**Figure 10:** CTL, NK, MA, DC, EP cell counts shown *in silico* immune simulation. **(A)** CD8 T-cytotoxic lymphocytes count, Total and memory shown; **(B)** CD8 T-cytotoxic lymphocytes count per entity-state; **(C)** Natural Killer cells (total count); **(D)** Epithelial cells, Total count broken down to acgive, virus-infected and presenting on class-I MHC molecule; **(E)** Macrophages. Total count, internalized, presenting on MHC class-II, active and resting macrophages; **(F)** Dendritic cells, DC can present antigenic peptides on both MHC class-I and class-II molecules, The curves show the total number broken down to active, resting, internalized and presenting the ag; Act, active; Intern, internalized the Ag; Pres II, presenting on MHC II; Dup, in the mitotic cycle; Anergic, anergic; Resting, not active.

**Figure 11:** Immunoglobulin and immune complex; Change trend of cytokines and interleukins. **(A)** Antigen and immunoglobulins, Antibodies are sub-divided per isotype (β-Defensin I molecular adjuvant including); **(B)** Antigen and immunoglobulins. Antibodies are sub-divided per isotype (β-Defensin I molecular adjuvant not including); **(C)** Concentration of cytokines and interleukins. Inset plot shows danger signal together with leukocyte growthfactor IL-2.

### 3.9. Computer simulation clones of candidate vaccines

The Gene infinity server conducted back translation of the vaccine construct. GenScript Tool was used for evaluating the gene sequence's key properties, including the Codon Adaptation Index (*CAI*) and GC content. The optimized nucleotide sequence *CAI* value was 1, and the GC content of the optimized sequence was 54.19% in *E. coli*. Recognition sites for *BamHI* and *XhoI* restriction enzymes were added to the optimized gene's 5' and 3' ends. The adapted codon sequence was inserted into the pET32a (+) vector using SnapGene software.

The article "Epitopes screening and vaccine molecular design of SADS-CoV based on immunoinformatics" was retracted in 2023. Reason: concerns about the authorship.

## 4. Discussion

Coronavirus had long been considered trivial pathogens, but the recent discovery of a new CoV strain officially named SARS-CoV-2 had sparked a deadly global COVID-19 pandemic (39). As the fourth recently discovered porcine enteric coronavirus, SADS-CoV of the same genus has successively hit several intensive pig farms and brought severe challenges to the prevention and control of swine diseases (40). The results of the metagenomic sequence of the SADS-CoV outbreak in 2019 showed that it had mutated and become more virulent, suggesting that early control and prevention of the epidemic had become necessary (41). However, although the current research results have made some progress in the origin, pathogenicity, diagnostic methods, and detection technologies of viruses, there are still many unsolved problems. For example, there was no report on the research progress of reliable drugs and vaccine preparation for this bat-derived coronavirus. Vaccination has always been an effective measure to prevent and control infectious diseases (42). Therefore, in order to prevent the continuous spread of SADS-CoV, there was an urgent need for effective vaccines. Immunoinformatics approaches have helped researchers predict and analyze potential epitopes needed to develop epitope vaccine candidates and screen the viral genome to identify immunogenic epitopes that elicit highly targeted immune responses without reversing the virus pathogenesis (43).

Based on this strategy, and to avoid excess antigen load and allergic reactions in the host, this study aims to design an candidate vaccine against SADS-CoV S protein so that the constructed candidate vaccine can generate humoral and cell-mediated immunity, thereby achieving immune balance. In addition to induced neutralized antibodies, the vaccine's protective effect also depends on cytotoxic CD8 T and helper CD4 T cells to eliminate the virus. One of the important features of immune response was the activation of helper T cell subtypes and releasing corresponding specific types of cytokines (44). The antigen epitope on MHC-II could activate Th1 and Th2 helper cells, and Th1 can release interference γ (IFN-γ), activate macrophages, and recognize and remove pathogens in cells. Helper T cells, Th2 mainly secrete cytokine interleukin 4 (IL-4), which could promote the proliferation and differentiation of antigen-presenting cells (18, 19). MHC-I restricted the transmission of pathogens by secreting unique antiviral cytokines and recognized and destroyed infected cells through the affinity between “antigenic peptide MHC” complexes, combined with proteasome processing and transporter associated with antigen processing (TAP) transport (45). Memory B cells can respond rapidly to recurred antigenic challenges and have more adaptive antibodies to prevent reinfection while contributing to immunity against homologous or heterologous viral infections (46). Therefore, ideal antigens should be presented by multiple MHC-I and MHC-II alleles and contain linear B cell epitopes related to neutralized antibodies (23). In order to enable animals to quickly cause immune response when they are attacked by SADS CoV again, and provide strong and lasting immune protection for them. The server recognizes the above epitope, but it was worth noting that the Th-5 epitope under the tertiary structure or the epitope is hidden and cannot be displayed. Fortunately, all epitopes are connected in a certain sequence through a flexible linker and introduced into β-defensin I construct epitope vaccine. The corresponding concept has also been used in the research and development of SARS CoV-2 candidate vaccine. From the selected dominant epitope regions, they are randomly distributed on the full length S protein without major concentration regions, which is consistent with previous research results (47). The selected flexible linkers also better avoid the generation of toxic side effects and improve the immune effect of the vaccine. The C-ImmSim server analysis showed that the candidate vaccine has good humoral and cellular immunity and the highest production of IFN-γ with a large amount of IL-10 and IL-2 activities. Excessive active immunoglobulins, IgM, IgG, and their possible involvement in isotype switch were also noted. Finally, the multi-epitope vaccine was codon-optimized, the *CAI* value was 1.0, and the GC content (54.19%) was also within the optimal limit, which indicated that the vaccine might be highly expressed in the *E. coli* K-12 system. SnapGene was used to clone into *E. coli* vector ensures that the candidate vaccine can be accurately translated and stably expressed in the prokaryotic expression vector pET-32a(+). In this study, a series of immunoinformatics tools were used to construct an effective vaccine against SADS-CoV, the candidate vaccine structure has been created. The interaction and binding mode between the receptor and the vaccine protein are stable and can produce immune response to SADS CoV. But experimental verification is still needed to evaluate the immunogenicity and safety of the designed and constructed candidate vaccine. Therefore, this study will next perform high-throughput cloning of the constructed candidate vaccine, express and purify the recombinant protein, immunize animals, and perform an immunological evaluation to ensure the true potential of the designed epitope vaccine against SADS-CoV.

The article "Epitopes screening and vaccine molecular design of SADS-CoV based on immunoinformatics" was retracted in 2023. Reason: concerns about the authorship.

## 5. Conclusions

This study successfully predicted and screened the dominant epitope of SADS-CoV S protein using the immunoinformatics method and constructed an candidate vaccine composed of CTL epitope, Th epitope, and linear B cell epitope that could trigger a strong immune response. This project will provide a new theoretical basis for designing SADS-CoV antiviral drugs and research on coronaviruses such as SARS-CoV-2.

## Data availability statement

The original contributions presented in the study are included in the article/supplementary material, further inquiries can be directed to the corresponding author.

## Author contributions

SL and YC came up with and designed the study. SL performed the experiments and wrote the manuscript. YC revised the manuscript. All authors contributed to the article and approved the submitted version.
